The article "Noninvasive Indirect Markers of Liver Fibrosis in Alcoholics" was published in 2019. Journal: Biomed Res Int.

# Noninvasive Indirect Markers of Liver Fibrosis in Alcoholics

**DOI:** 10.1155/2019/3646975

**Published:** 2019-05-05

**Authors:** Lech Chrostek, Dagmara Przekop, Ewa Gruszewska, Monika Gudowska-Sawczuk, Bogdan Cylwik

**Affiliations:** ^1^Department of Biochemical Diagnostics, Medical University of Bialystok, Waszyngtona 15A, 15-269 Bialystok, Poland; ^2^Department of Pediatric Laboratory Diagnostics, Medical University of Bialystok, Waszyngtona 17, 15-274 Bialystok, Poland

## Abstract

The aim of this study was to evaluate the diagnostic values of noninvasive indirect markers of liver fibrosis: APRI, GAPRI, Forns, FIB-4, Age-Platelet, and Hepascore in alcoholics. Blood samples were collected from a randomized group of 142 alcohol-dependent patients. The diagnosis of dependency was made according to the ICD-10 WHO criteria. The values of noninvasive markers were calculated with specific algorithms. The fibrosis stage was evaluated on the basis of FibroTest. The values of APRI, Forns, FIB-4, GAPRI, AP, and Hepascore differ between various stages of liver fibrosis. Patients with fibrosis stage F0 present lower values of APRI, Forns, FIB-4, GAPRI, and Hepascore in comparison to the patients with stages F1 and F0-F1. Patients with fibrosis stages < F2 have lower values of all noninvasive markers than patients with stages ≥F2. Patients with fibrosis stages ≥F2 but <F4 have lower values of APRI, Forns, FIB-4, GAPRI, and Hepascore than patients with stage F4. The values of noninvasive markers tested here differ in various stages of liver fibrosis. To our surprise, the patented marker, Hepascore, achieves a lower diagnostic value in alcoholics than simple markers involving only liver enzymes, platelet count, and cholesterol. The best marker of liver fibrosis in alcoholic patients seems to be the Forns index.

## 1. Introduction

Liver diseases induced by excessive alcohol consumption are an important cause of morbidity and mortality worldwide. Alcoholic liver diseases (ALD) can manifest themselves as a one of the following disorders: alcoholic fatty liver, alcoholic hepatitis, and alcohol-related cirrhosis [1, 2]. The studies have shown that the alcoholic liver injury can develop into fibrosis or cirrhosis in up to 15% of alcoholics [3, 4]. On the other hand, alcoholic hepatitis and steatohepatitis are present in 35% of alcoholics [5]. Therefore, detection of an early stage of liver damage is the key to provide a positive outcome for therapeutic intervention. The “gold standard” for evaluating the stage of liver fibrosis—liver biopsy—is an invasive procedure which can lead to health complications in 3.0% of patients (e.g., bleeding, pain, bile peritonitis, kidney puncture, or death). Additionally, sampling errors are very common due to difficulty with obtaining liver specimen representing the whole liver [6–8]. Therefore, there is a great need for developing safer and freely available noninvasive diagnostic tools. In this study, we will follow the work of Thiele et al. who compared the accuracy of 10 liver fibrosis markers (patented or not) in patients with alcoholic liver diseases [9]. According to these results, the receiver operating characteristic curve (AUROC) of two tests—ELF and FibroTest—for advanced fibrosis (≥F3) reached and exceeded the value of 0.9. Taking into account the fact that, among others, these two tests exhibited the highest diagnostic power for identification of alcoholic patients with advanced liver fibrosis, we have treated the FibroTest as a matrix for comparing the diagnostic values of five nonpatented, noninvasive indirect markers of liver fibrosis: APRI, GAPRI, Forns, FIB-4, Age-Platelet (AP), and one patented algorithm, Hepascore, in alcoholics. Additionally, carbohydrate-deficient transferrin (CDT) as an established marker of alcohol abuse was evaluated in these patients [10]. According to our previous published work, the relative values of CDT are affected by liver diseases and reflected the severity of liver dysfunction [11].

## 2. Materials and Methods

### 2.1. Participants

The tested group consisted of 142 alcohol-dependent patients (127 men and 15 women) from detoxification ward (Department of Detoxification, Psychiatric Hospital in Choroszcz). Patients were initially examined and interviewed regarding history of disease and their use of alcohol. The diagnosis of dependency was made on the basis of ICD-10 WHO criteria. The self-reported mean alcohol consumption was 1311 g of ethanol per week and mean time of dependency was 18 years. The patients did not undergo the liver biopsy, and fibrosis stage was established in FibroTest which was used as the reference standard. Study was in accordance with Helsinki Declaration and was approved by the Bioethical Committee at the Medical University in Bialystok.

### 2.2. Blood Sampling

Blood samples from a peripheral vein from each patient were collected. After centrifugation, sera were collected into 2 tubes and stored at -86°C until assayed. Besides serum, a part of each sample was collected into tubes containing 3.8% liquid sodium citrate and EDTA-2.

AST, ALT, GGT, cholesterol, *α*2-macroglobulin, hyaluronic acid, and bilirubin were determined on the Architect c8000 (Abbott Laboratories, Abbott Park, USA). PLT count was measured on Sysmex XS-800i (Sysmex Corporation, Singapore).

The serum biochemical markers, *α*2-macroglobulin, haptoglobin, apolipoprotein A1, *γ*-glutamyltransferase, alanine aminotransferase, and total bilirubin, were determined according to methods recommended by BioPredictive (Paris, France). FibroTest scores were computed by BioPredictive company according to the arrangement, and results were provided with security algorithms.

CDT immunoassays were carried out using the N Latex CDT test (Siemens Healthcare Diagnostics, Marburg, Germany) on BN II System (Siemens Healthcare Diagnostics, USA). CDT values were expressed as percentages of total transferrin.

### 2.3. Calculations

(1) APRI=ASTIU/L/50IU/LPLT109/L∗100GAPRI=GGTIU/LPLT109/L∗100FIB-4=age∗ASTIU/LPLT109/L∗√ALTIU/LForn's  index=7.811−3.131ln⁡PLT109/L+0.781ln⁡GGTIU/L+3.467ln⁡age−0.014cholesterolmg/dLAP  index=age+PLTage: <30=0;  30-39=1;  40-49=2;  50-59=3;  60-69=4;  ≥70=50,PLT×109/L
: ≥225=0;  200-224=1;  175-199=2;  150-174=3;  125-149=4;<125=5Hepascore=Y1+YY=exp-4.185818−0.0249∗age+0.7464∗sex+1.0039∗α2-macroglobulin+0.0302∗hyaluronic  acidng/mL+0.0691∗total  bilirubin–0.0012∗GGT  IU/L

The values for sex: 1 for men and 0 for women.

### 2.4. Statistical Analysis

The normality of distribution was checked by means of Kolmogorov-Smirnov test with the Lilliefors correction. The analysis revealed that the distribution of APRI, FIB-4, GAPRI, and Hepascore does not follow a normal distribution (P<0.05), but Forns index and AP follow a normal distribution (p>0.05) (Figure 1). The differences between stages of liver fibrosis were evaluated by Mann-Whitney U test. To test the effect of liver diseases on the values of markers, ANOVA rank Kruskal-Wallis test was performed. We considered* P-*values <0.05 as statistically significant. The diagnostic performance of each test was calculated as sensitivity, specificity, PPV, NPV, and accuracy. To calculate the diagnostic accuracy of algorithms, the ROC curve was used.

## 3. Results

The average values of noninvasive markers in patients with different liver fibrosis scores are presented in Table 1. The values of APRI, Forns, FIB-4, GAPRI, AP, and Hepascore differed between the stages of liver fibrosis (ANOVA rank Kruskal-Wallis test: H=30.902, P<0.001; H=49.386, P<0.001; H=51.907, P<0.001; H=40.951, P<0.001; H=31.553, P<0.001; H=46.019, P<0.001, respectively). The levels of CDT were similar in all stages of liver fibrosis (H=13.243, P=0.066), but %CDT values were different (H=13.948, P=0.050). Patients with no or mild fibrosis (F0, F0-F1, F1, F1-F2) had lower values of all noninvasive markers than patients with moderate, advanced, or severe fibrosis (F2, F3, F3-F4, F4) (P<0.001 for all comparisons). Then, patients with fibrosis stages F2, F3, and F3-F4 had lower values of APRI, Forns, FIB-4, GAPRI, and Hepascore than patients with cirrhosis (F4) (P=0.038, P=0.017, P=0.024, P=0.012, P=0.035, respectively). We also observed that patients with no fibrosis (F0) had lower values of APRI, Forns, FIB-4, GAPRI, and Hepascore in comparison to patients with mild fibrosis (F0-F1 and F1) (Mann-Whitney U test: P=0.030, P=0.002, P=0.044, P=0.001, P=0.039, respectively). The values of AP index were similar in fibrosis stages F0, F0-F1, F1 (P=0.089) and F2, F3, F3-F4, F4 (P=0.173).

The average values of APRI, Forns, FIB-4, GAPRI, AP, and Hepascore were significantly higher in patients with cirrhosis (F4) in comparison with patients without fibrosis (F0) (P<0.001, P<0.001, P<0.001, P<0.001, P=0.002, P<0.001, respectively). In addition, the values of FIB-4 and GAPRI in fibrosis stage F4 were higher than those in stage F0-F1 (P=0.005, P=0.018, respectively), and Hepascore in fibrosis stage F4 was higher compared to the stage F1 (P=0.004). The average value of GAPRI in fibrosis stage F4 was also higher than the one in the stage F1-F2 (P=0.025), and in the stage F3 it was higher than in the stage F0 (P=0.038). Hepascore, AP, and Forns scores were higher in patients with the stage F2 than in patients with the stage F0 (P=0.027, P=0.004, P=0.026, respectively). %CDT was lower in patients with advanced fibrosis/cirrhosis than in those with the stage F2 (P=0.011).

Three out of seven markers, GAPRI, Hepascore, and FibroTest, exhibited significantly higher results in patients with significant fibrosis (F≥2) in comparison to those with no significant fibrosis (F0-F1, F1, F1-F2), but all tested markers had higher values in patients with cirrhosis (F3-F4, F4) when compared to those without cirrhosis (F0-F1, F1, F1-F2, F2, F3) (Table 2).

Diagnostic power of liver fibrosis markers is presented in Table 3. Our study has shown that Forns index reached an ideal diagnostic accuracy (of 100%) and an ideal diagnostic power (AUC=1.0) for fibrosis detection in alcoholics. The remaining tests exhibited a high diagnostic power (AUCs over 0.9 for all with the exception of AP index) in the detection of fibrosis in alcoholic patients. We could observe that tested markers, except for Forns index, exhibited a high diagnostic specificity and positive predictive value (PPV). The markers APRI, GAPRI, and FIB-4 had similar diagnostic values (sensitivity: above 80%, specificity: 95% and above, accuracy: above 80%, PPV: above 99%, NPV: above 40%, and AUCs: above 0,930). Hepascore has shown a lower diagnostic accuracy (ACC<80%) than simple markers (FIB-4, Forns, GAPRI, and APRI).

Spearman's rank test demonstrated that there was a correlation between APRI, Forns, FIB-4, GAPRI, AP, Hepascore, and FibroTest in alcoholic patients (P<0.001 for all comparisons), but there was no correlation between CDT, %CDT, and FibroTest (P=0.468, P=0.556, respectively) (Figure 2).

## 4. Discussion

The evaluation of the severity of liver fibrosis and the associated inflammation is crucial for determination of therapeutic strategies, prognosis, and predicting potential complications in patients with alcoholic liver diseases [12]. An ideal noninvasive marker for the assessment of fibrosis in ALD should accurately and with high diagnostic sensitivity detect the presence of fibrosis as well as evaluating the stage of liver fibrosis. One of the most widely used patented liver fibrosis marker, FibroTest, has been validated in patients with hepatitis C, hepatitis B, nonalcoholic steatohepatitis, and alcoholic liver diseases [13–16]. It combines five biochemical serum markers (*α*2-macroglobulin, haptoglobin, *γ*-glutamyltransferase, bilirubin, and apolipoprotein A1) with patient's age and gender [16]. In the last large meta-analysis, FibroTest showed a good diagnostic accuracy for significant fibrosis (≥F2) and cirrhosis (F4) without discriminating between chronic liver diseases of different etiologies (mean standardized AUC for significant fibrosis was 0.84) [17]. Result of FibroTest reflects fibrosis stages according to the most used histological classification, METAVIR scoring system [18]. In our study the severity of liver damage was diagnosed on the basis of FibroTest. According to American College of Gastroenterology guidelines for alcoholic liver disease, “liver biopsy is not routinely recommended for diagnosis of alcoholic fatty liver disease. However, liver biopsy and noninvasive tools of fibrosis may be considered for diagnosis of steatohepatitis and/or liver fibrosis.” [19]. The prospective study confirms the good diagnostic value of biochemical tests for fibrosis as compared with the histological analysis of liver biopsy with special caution FibroTest results with significant elevation of ALT, and/or GGT, and/or alpha-2-macroglobulin [20]. EASL Clinical Practical guidelines recommend liver biopsy for histological diagnosis of ALD [21]. According to these, liver biopsy can be done percutaneously in most patients and requires a transjugular approach in patients with a low platelet count and/or a prolonged prothrombin time. Additionally, liver biopsy is an invasive procedure with significant morbidity. Therefore, EASL guidelines do not recommend it for all patients with suspected ALD. We are aware that liver biopsy is considered as a gold standard for staging and grading of liver fibrosis but there are discordance between the degree of liver injury estimated by liver biopsy and that estimated by a panel biochemical markers. The main difficulty in this discordance analysis was the absence of a true reference standard for liver injury. The two main causes of failure for biopsy are sampling error and observer error. Poynard and coworkers stated that they “never made a management decision based on biopsy results for the following other causes: alcohol abuse, steatohepatitis, drug-induced liver disease, hemochromatosis or coinfection with hepatitis B virus or HCV.” [22]. False-positive results for fibrosis based on FibroTest scores occurred in only hundredth of patients in the hospital based cohort and were attributable to various causes. It can be Gilbert syndrome (an increase in unconjugated bilirubin), hemolysis (an increase in unconjugated bilirubin and a decrease in haptoglobin), and acute inflammation (an isolated increase in *α*2-macroglobulin [22].

In this study, we have compared the diagnostic values of simple, noninvasive liver fibrosis markers in alcoholics. First, specificity of 100% and PPV of 100% for APRI, GAPRI, Forns index, and Hepascore have been noted. It means that there were no false-positive results in nonalcoholic patients. However, this excellent specificity was not accompanied by the highest sensitivity. It means that false negative results were present in alcoholic patients. The low negative predictive value of all markers, with the exception of Forns index, derived also from the high number of false negative results in alcoholics. It is clear that the cut-off points indicated by ROC curve are more shifted to lower values than indicated in literature data. For example, cut-off point of APRI for differentiation between no/significant/advanced fibrosis (from stage F0 to stage F3) and cirrhosis (F4) taken from literature equals 2.00, but in our study it is 0.34 [23]. The cut-off point of Hepascore for differentiation between stages F0-F2 and F3-F4 obtained the value of 0.50, but in our study it is only 0.20 [24]. The discriminative point for FIB-4 between no fibrosis and advanced fibrosis (F3-F4) was assigned to the value of 3.27, but cut-off point from ROC curve in this study reached the value of 1.24 [25]. Only the cut-off point for Forns index discriminating no fibrosis from advanced fibrosis (F≥3) equal to 4.20 was similar to the cut-off point in our study [26].

The fine specificity and PPV for APRI and GAPRI might be the result of these markers accounting only for liver enzymes (AST or GGT) and platelet count. Forns index additionally includes cholesterol, but reached an absolute diagnostic power. The level of cholesterol decreases significantly with the degree of fibrosis progression and, therefore, can reflect the degree of impairment of liver function. [27]. A score below 4.2 excluded significant fibrosis in patients with chronic hepatitis C with accuracy of 96% [26]. Forns et al. demonstrated that this model is not sufficient to detect significant fibrosis, because of its 66% positive predictive value. Thiele et al. presenting biopsy-controlled study indicated Forns index as the best performing indirect index of advanced fibrosis [9]. On the other hand, FIB-4 based on both aminotransferases level and platelet count did not reach ideal diagnostic values. It is well established that aminotransferases (ALT and AST) constitute a part of standard laboratory panels examined in patients with liver diseases and that the most specific liver enzyme is alanine aminotransferase [28]. In turn, elevated number of platelets is a common complication in patients with chronic liver disease (PLT <150 x 10^9^/L) [29]. According to the published data, the value of APRI index over 1.5 accurately predicts significant fibrosis (AUC=0.88) and the value over 2.0 cirrhosis (AUC=0.94) in patients with chronic HCV [23]. APRI also correlated with the stage of fibrosis more strongly than AST or PLT alone. The next noninvasive marker of liver fibrosis tested, FIB-4, includes PLT count in addition to aminotransferases [25]. The FIB-4 score of ≥3.25 allows for a correct identification of patients who have significant fibrosis and could avoid liver biopsy. The values of FIB-4 ≥1.45 and ≥3.25 showed a good concordance with FibroTest (92.1% and 76%, respectively).

In our study, the values of all tested markers differed between stages of liver fibrosis. It is noteworthy that the majority of markers (except AP) allow differentiating between no fibrosis (F0) and mild fibrosis (F0-F1 and F1). In addition, patients with no, minimal, and mild fibrosis (F0, F0-F1, F1, F1-F2) had lower values of all markers than patients with moderate, advanced, or severe fibrosis/cirrhosis (F2, F3, F3-F4, F4). Finally, patients with the stages F2, F3, and F3-F4 fibrosis had lower values of markers (excluding AP) than patients with cirrhosis (F4). Secondly, we have shown that the markers APRI, GAPRI, and FIB-4, which incorporate liver enzymes (ALT, AST, GGT, and PLT), obtained similar diagnostic sensitivity, specificity, accuracy, PPV, NPV, and AUCs. The more complicated marker (Hepascore) had a lower diagnostic accuracy (ACC<80%) than simple markers (FIB-4, Forns, GAPRI, and APRI). This can be explained by the lower diagnostic sensitivity of this test (<80%). The imprecision of the determinations of multiple components should also be taken into consideration. However, adding cholesterol and platelet count to Forns index maximizes diagnostic values. Adding further tests to the algorithms decreases their diagnostic values, which is visible in the example of Hepascore.

Platelet counts and age are required to calculate the AP index. According to the study of Poynard and Bedossa, platelet count and age of patients are factors independently correlated with the presence of fibrosis and histological activity of liver disease [30]. With cut-off value of 6.0 or greater, the AP index diagnoses significant fibrosis with sensitivity of 52% and specificity of 93%. In our study, at the cut-off point of 4.0, we have obtained a similar sensitivity of 61.3% and specificity of 93.9%. The AP index demonstrated a lower diagnostic power to predict fibrosis in alcoholic patients.

The patented algorithm Hepascore combines the results obtained from the following biochemical tests: bilirubin, GGT, *α*2-macroglobulin, and hyaluronic acid [31]. Hepascore values of ≥0.50 can predict significant fibrosis with the specificity of 89%–92%. We have obtained cut-off point for Hepascore equal to 0.20, which is lower than that reported by Adams and coworkers [31]. A big advantage of Hepascore is the fact that GGT and bilirubin are measured routinely and *α*2-macroglobulin can be determined in any laboratory with a nephelometer using commercially available antibodies. The last parameter included in Hepascore, hyaluronic acid, is considered as a direct marker of liver fibrosis, as its synthesis is associated with the deposition of extracellular matrix [32]. It was found that serum levels of hyaluronic acid are elevated in chronic liver diseases in which the serum levels of ECM are also changed [33].

Carbohydrate-deficient transferrin (CDT) is one of the most used biomarkers of chronic alcohol abuse, mainly because of its high specificity [10]. However, the diagnostic efficiency of CDT as a marker of chronic alcohol abuse is diminished by its low diagnostic sensitivity. There are many clinical conditions that can affect the number of false-positive results in healthy controls. One of them is advanced liver diseases such as liver fibrosis and hepatocellular carcinoma [34]. According to these data the results of CDT are similar in patients with alcoholic cirrhosis and controls without liver diseases. Our alcoholic patients with cirrhosis (stage F4) have lower relative CDT values than alcoholics without fibrosis (stage F0). All tested fibrosis markers (APRI, Forns index, FIB-4, GAPRI, AP, and Hepascore) obtained higher results in stage F4 than in stage F0. It is necessary to mention here that alcoholics with score A cirrhosis (Child-Pugh scale) reached similar results of %CDT to the values in the healthy controls [11]. In this work the values of %CDT were different in the stages of liver fibrosis and were the highest in the advanced fibrosis (stage F2) and the lowest in alcoholic cirrhosis (stage F4). According to that we can conclude that the end stage of liver fibrosis diminished the sensitivity of CDT as a marker of chronic alcohol abuse, which is consistent with our previous study.

## 5. Conclusion

Our results suggest that simple blood tests incorporated in complex markers can be helpful in identifying a specific stages of liver fibrosis. Surprisingly, the patented algorithm, Hepascore, shows a lower diagnostic value in randomized group of alcoholics than simple markers involving only liver enzymes, platelet count, and cholesterol. According to our data the best marker of liver fibrosis in alcoholic patients is the Forns index.

## Figures and Tables

**Figure 1:** The distribution of noninvasive markers of liver fibrosis in alcoholics.

**Figure 2:** Spearman's rank correlation between tested noninvasive liver fibrosis markers and FibroTest.

**Table 1:** The values of noninvasive markers according to stages of liber fibrosis.

Marker	FibroTest score						
	F0 (n=52)	F1 (n=8)	F1-F2 (n=28)	F2 (n=11)	F3 (n=8)	F3-F4 (n=2)	F4 (n=12)
APRI	0.91±1.10	2.68±2.56	1.80±1.72	1.77±1.57	1.73±1.67	6.20±1.57	3.66±2.62
Forn's	7.31±1.68	9.38±1.44	9.10±1.92	9.89±1.66	8.96±1.32	12.97±1.14	11.50±1.79
FIB-4	2.60±2.24	5.20±3.04	4.72±3.92	6.60±6.28	3.60±1.94	17.20±7.72	9.69±4.65
GAPRI	58.90±85.34	164.67±101.30	187.55±279.82	175.29±152.20	320.66±333.47	858.87±20.00	827.54±709.34
AP	3.44±2.02	5.25±1.83	5.00±2.24	6.00±1.94	4.38±2.00	8.00±0.00	6.67±2.42
Hepascore	0.25±0.13	0.28±0.17	0.42±0.21	0.59±0.28	0.59±0.32	0.70±0.28	0.82±0.20
CDT	114.69±60.97	119.80±73.27	114.91±66.20	157.25±60.99	82.86±33.03	93.85±3.18	72.26±39.51
%CDT	4.38±2.60	5.55±3.92	5.14±3.35	7.23±2.49	3.62±1.75	4.72±0.45	2.95±1.60

Data are presented as mean ± SD.

**Table 2:** The values of noninvasive markers in patients with significant, no significant fibrosis, without and with cirrhosis.

Fibrosis Markers	No significant fibrosis (F0-F1, F1, F1-F2) (n=51)	Significant fibrosis (F≥2) (n=21)	Without cirrhosis (F0-F1, F1, F1- F2, F2, F3) (n=76)	Cirrhosis (F3-F4, F4) (n=14)
APRI	1.72 ± 1.73	2.18 ± 2.21	1.80 ± 1.74	4.02 ± 2.84
		P1=0.254		P2=0.001*∗*

Forn's	8.85 ± 1.79	9.83 ±1.83	9.12 ± 1.92	11.71 ± 1.77
		P1=0.063		P2<0.001*∗*

FIB-4	4.21 ± 3.37	6.47 ± 6.23	4.64 ± 4.01	10.77 ± 5.50
		P1=0.131		P2<0.001*∗*

GAPRI	158 ± 219	295 ± 300	276 ± 287	832 ± 652
		P1=0.020*∗*		P2<0.001*∗*

AP	4.74 ± 2.27	5.57 ± 2.13	4.91 ± 2.23	6.86 ± 2.28
		P1=-1.003		P2=0.004*∗*

Hepascore	0.39 ± 0.21	0.60 ± 0.28	0.43 ± 0.25	0.80 ± 0.21
		P1=0.008*∗*		P2<0.001*∗*

FibroTest	0.32 ± 0.08	0.58 ± 0.08	0.38 ± 0.14	0.87 ± 0.09
		P1<0.001*∗*		P2<0.001*∗*

Data are presented as mean ± SD. P1: P value between significant and no significant fibrosis; P2: P value between cirrhosis and no cirrhosis; *∗* means statistically significant difference.

**Table 3:** Diagnostic value of liver fibrosis markers in alcoholics.

Marker	Cut-off	Sensitivity [%]	Specificity [%]	ACC [%]	PPV [%]	NPV [%]	AUC± SE
FIB-4	1.24	85.8	95.0	87.0	99.2	48.7	0.948±0.018
Forn's	4.11	100	100	100	100	100	1.0 ± 0.0
Hepascore	0.20	75.8	100	79.2	100	40.0	0.942±0.02
GAPRI	20.07	81.6	100	83.9	100	43.5	0.931±0.02
APRI	0.34	81.6	100	83.9	100	43.5	0.934±0.02
AP	4.00	64.5	90.0	67.7	97.8	26.5	0.867±0.036
FibroTest	0.21	61.3	93.9	69.9	96.6	46.5	0.795±0.031

## Data Availability

The data used to support the findings of this study are available from the corresponding author upon request.
